# Correlation of Inpatients Suffering from Acute Acalculous Cholecystitis during ICU Treatment with Acute Physiology and Chronic Health Evaluation II Score, Duration of Ventilator Use, and Time on Total Parenteral Nutrition

**DOI:** 10.1155/2022/3407997

**Published:** 2022-06-30

**Authors:** Yunfeng Zhang, Kaixian Wang, Yuhui Wang, Yang Liu

**Affiliations:** Department of Critical Care Medicine, Tangshan Workers Hospital, Tangshan, 063000 Hebei, China

## Abstract

**Objective:**

To explore the correlation of inpatients suffering from acute acalculous cholecystitis (AAC) during ICU treatment with Acute Physiology and Chronic Health Evaluation II (APACHE-II) score, duration of ventilator use, and time on total parenteral nutrition (TPN).

**Methods:**

From March 2016 to March 2022, the clinical data of 47 patients with AAC who received ICU treatment in our hospital were retrospectively reviewed, and these patients were included in the AAC group. Another 36 patients treated in the ICU in the same period with age and gender matching with those in the AAC group were selected as the non-AAC group. Patients' various clinical data were recorded to analyze the correlation of AAC with APACHE-II score, duration of ventilator use, and time on TPN.

**Results:**

The shock time, duration of ventilator usage, and duration of sedative medicine use were all substantially longer in the AAC group than in the non-AAC group, according to the univariate analysis (*P* < 0.05); the amount of norepinephrine used, white blood cell count, C-reactive protein (CRP) amount, and APACHE-II score were significantly higher in the AAC group than in the non-AAC group (*P* < 0.05); between the two groups, the time on TPN and fasting time were different, but with no statistical significance (*P* > 0.05); after performing Spearman's correlation with the significantly between-group different indicators, the result showed that the amount of norepinephrine used, duration of ventilator use, white blood cell count, and CRP amount were significantly correlated with the occurrence of AAC, and the correlation was positive (*P* all <0.001).

**Conclusion:**

The APACHE-II score and time on TPN are not significantly correlated with the occurrence of AAC; and the amount of norepinephrine used, duration of ventilator use, white blood cell count, and serum CRP are positively correlated with the occurrence of AAC. Measuring the variations in the levels of various markers can signal the onset of AAC or reflect the state and prognosis, suggesting a possible application in clinic-based targeted prevention and treatment of AAC.

## 1. Introduction

Acute acalculous cholecystitis (AAC) is a clinical emergency with lower morbidity, which tends to occur in critically ill patients with severe trauma, burns, shock, hypotension, or after major surgery, is featured with insidious onset, atypical clinical presentation, and rapid progression of the condition, and easily causes perforated gangrene and other complications, leading to a high clinical mortality [1–4]. Most patients treated in ICU inpatient areas are critically ill with complex condition and often accompanied by multivisceral dysfunction, so they are at high risk for AAC; in addition, patients who undergo the therapeutic means such as sedation and mechanical ventilation often have disorders of consciousness, and thus, the condition of AAC is not easily perceived, resulting in a prolonged disease course and a high clinical mortality rate of 45-50% [5–8]. To enable clinicians to better monitor patients' gallbladder changes, control patients' conditions, and realize early detection, diagnosis, and treatment of AAC, a detailed analysis of each risk factor that can easily trigger AAC is required.

Many reports on AAC in recent years have shown that the incidence of AAC is clearly increasing, not only in critically ill patients like trauma and burns but also in patients with basic diseases like diabetes, hypertension, chronic bronchitis, and systemic lupus erythematosus, and that the disease group is becoming younger and younger [9–11]. However, the current published works on AAC in China are focused on disease diagnosis and treatment and technology update, promoting the development of curation, but there are few reports on analyzing the risk factors triggering AAC. To explore the factors that contribute to the development of AAC in critically ill patients, the study retrospectively analyzed the patients treated in our ICU to reduce their length of stay in the ICU and lower the case fatality rate of AAC in ICU patients.

## 2. Materials and Methods

### 2.1. Selection of Study Subjects in the AAC Group

1. The patients were ICU inpatients and treated in ICU for more than 24 h
2. The patients met the diagnosis criteria for AAC [12]
3. The patients were clearly diagnosed with normal gallbladder on admission and then were diagnosed with AAC during ICU treatment
4. The patients were at least 18 years old
5. The patients did not have severe cirrhosis, liver failure, acute leukemia, and other diseases
6. The patients were confirmed to have no cholecystolithiasis and choledocholith after imaging examination
7. The patients did not have the history of cholecystectomy
8. The patients had complete clinical data
9. The patients and their family members understood the study and signed the informed consent

Finally, 47 AAC patients who were treated in our hospital from March 2016 to March 2022 and met the study criteria were selected as the AAC group.

### 2.2. Selection of Study Subjects of the Non-AAC Group

1. The patients were treated in the ICU in the same period with age and gender matching with those in the AAC group
2. The patients did not have AAC during ICU treatment

The clinical data of 36 non-AAC patients were selected for the retrospective analysis study and set as the non-AAC group.

### 2.3. Ethical and Moral Standards

The study plan was reviewed, approved, and monitored by the Hospital Ethics Committee; and the ethical and moral standards met the World Medical Association Declaration of Helsinki (2013) [13].

### 2.4. Study Contents

#### 2.4.1. General Data

The age, body mass index (BMI), gender, length of hospital stay, smoking, drinking, nationality, place of residence, and other general data of patients in the two groups were recorded to clarify the balance and comparability of the two groups by statistical analysis.

#### 2.4.2. Clinical Data

Based on the early data analysis and summary of previous studies, the risk factors that might cause AAC were used for further between-group comparison and analysis, including the shock time, amount of noradrenaline used, duration of ventilation use, white blood cell count, C-reactive protein (CRP), the Acute Physiology and Chronic Health Evaluation II (APACHE-II) score, time on total parenteral nutrition (TPN), length of sedative medication use, and fasting time.

#### 2.4.3. Correlation Analysis

To clarify the association between each metric and AAC, the above indicators that showed significant differences were subjected to correlation analysis using the statistical tool Spearman. Spearman's rank correlation coefficient is a nonparametric measure of the dependency of two variables, and the correlation of two statistical variables was evaluated using a monotonic equation.

### 2.5. Statistical Processing

In this study, the data processing software was SPSS 22.0, which was mainly used to calculate the between-group differences of data, the picture drawing software was GraphPad Prism 7 (GraphPad Software, San Diego, USA), the items included were enumeration data and measurement data, which were expressed by [*n* (%)] and ($\bar{x}\pm s$) and examined by *X*^2^ test and *t*-test, respectively, and met normal distribution, and between-group differences were considered statistically significant at *P* < 0.05.

## 3. Results

### 3.1. General Data

The patients' age, BMI, gender, length of hospital stay, smoking, drinking, nationality, place of residence, and other general data were not statistically different between the two groups (*P* < 0.05), presenting comparability. See Table 1 for the specific data.

### 3.2. Clinical Data

The shock time, duration of ventilator use, and duration of sedative medication use were significantly longer in the AAC group than in the non-AAC group (*P* < 0.05); the amount of norepinephrine used, white blood cell count, CRP amount, and APACHE-II score were significantly higher in the AAC group than in the non-AAC group (*P* < 0.05); between the two groups, the time on TPN and fasting time were different, but with no statistical significance (*P* > 0.05). See Table 2.

### 3.3. Correlation Analysis

After performing Spearman's correlation with the significantly between-group different indicators, including the amount of norepinephrine used, duration of ventilator use, white blood cell count, CRP amount, APACHE-II score, and duration of sedative medication use, it was found that the amount of norepinephrine used, duration of ventilator use, white blood cell count, and CRP amount were significantly correlated with the occurrence of AAC, and the correlation was positive (*P* all <0.001). See Table 3 for details.

## 4. Discussion

In contrast to calculous cholecystitis, AAC has an urgent onset, atypical symptoms, and rapid disease progression and is often accompanied by severe complications such as gangrene of gallbladder, perforation of gallbladder, and peritonitis, making it one of the important causes of death in patients [14–16]. Most ICU patients are acutely and critically ill with multiple organ dysfunction, making them vulnerable to AAC. These patients are unable to express their symptoms on their own, which, when combined with pharmaceutical interventions, examination limitations, and other factors, leads to delayed diagnosis and treatment, resulting in a high clinical mortality rate for AAC patients [17–20]. In recent years, increasing attention has been paid to AAC in clinic to clarify the potential pathogenic factors of AAC, and the development of targeted preventive measures for patients at high risk of AAC is urgent. However, current published works on AAC mostly focus on disease diagnosis and treatment, and there are still few studies on risk factors and correlation of AAC incidence. Based on this, a study of 83 patients admitted to our ICU ward was conducted with the aim of investigating common risk factors predisposing to AAC and the correlation between the occurrence of AAC and APACHE-II score, duration of ventilator use, and time on TPN. Clinical data from 44 patients were collected early in the investigation for a small retrospective analysis, and the link of parameters including shock duration, norepinephrine dose, and ventilator use with the development of AAC in ICU patients was studied for the first time herein.

After further expanding the sample size, it was concluded that according to the univariate analysis, the shock time, duration of ventilator use, and duration of sedative medication use were significantly longer in the AAC group than in the non-AAC group (*P* < 0.05); the amount of norepinephrine used, white blood cell count, CRP amount, and APACHE-II score were significantly higher in the AAC group than in the non-AAC group (*P* < 0.05); and between the two groups, the time on TPN and fasting time were different, but with no statistical significance (*P* > 0.05), which was consistent with the previous studies [21]. With further analysis, the following can be concluded. (1) Patients with shock are more prone to develop AAC, according to some published studies, because vasodilation and improved blood flow result in the reperfusion of blood with many inflammatory mediators, causing gallbladder injury and increasing gallbladder inflammation. In the univariate analysis of the study, the shock time was significantly different between the two groups, but it was not observed by Spearman's correlation, and it may be that the evaluation of shock time in patients was biased by drug treatment, and in such cases, gallbladder monitoring in shock patients should be enhanced in the clinic, and follow-up studies with larger sample size are required for verification.

(2) Norepinephrine is one of the common drugs to correct shock and a necessary drug for patients in ICU to maintain blood pressure and ensure blood supply to important organs. High dosages of norepinephrine will increase peripheral vascular resistance, constrict the flow of blood vessels to the gallbladder, create gallbladder blood supply problems and mucosal ischemia, and worsen gallbladder inflammation. Spearman's correlation analysis showed that norepinephrine dosage was positively associated with AAC, indicating that norepinephrine dosage is an important risk factor contributing to the development of AAC, and therefore, for ICU patients who need elevation of blood pressure by drugs such as norepinephrine, dynamic monitoring of their gallbladder should be enhanced to facilitate early detection of AAC and to apply targeted control measures.

(3) Although sedation and analgesia are important therapeutic linkages for ICU patients and are advantageous to their early recovery, sedative medicines have unavoidable side effects, such as gastrointestinal depression. Decreased gastrin can directly lead to insufficient secretion of cholecystokinin, failure of normal contraction of the gallbladder, bile retention in the gallbladder, absorption of bile water by gallbladder epithelial cells, and viscous bile that is difficult to excrete, causing cholestasis and aggravating damage to the gallbladder mucosa and proinflammatory reactions. Spearman analysis indicated that there was no significant correlation between the sedative drug dosage and AAC, which may be related to some factors such as patients' dosage difference and sample size.

(4) Assisted breathing by mechanical ventilation can cause increased intra-abdominal pressure, while continuous intra-abdominal hypertension can affect the blood supply to the intestine, causing ischemia and hypoxia of the intestinal mucosa and mucosal necrosis and sloughing and disrupting the intestinal mucosal barrier; in addition, continuous increased pressure in the abdominal cavity can also promote the passage of bacteria through the lymphatic system or blood into the biliary tract, causing bacterial infection in the gallbladder. Spearman's correlation analysis showed that the duration of ventilator use was positively correlated with AAC and was a significant risk factor for inducing AAC, so close attention should be paid to ICU patients receiving continuous mechanical ventilation in clinical treatment, so as to monitor gallbladder changes and prevent AAC occurrence.

(5) White blood cell count is an important observation indicator in cholecystitis patients, and this study confirmed that white blood cell count was positively associated with the occurrence of AAC. It is because individuals with AAC frequently have necrosis and perforation of the gallbladder wall, and gallbladder inflammation can quickly disseminate to the abdominal cavity, causing localised or diffuse peritonitis. Therefore, white blood cell count can be used as an important indicator to monitor changes in the gallbladder in ICU patients to suggest the lesion.

(6) CRP is one of the systemic inflammatory indicators for monitoring cholecystitis and a highly sensitive protein produced by the human liver, which is significantly higher in the acute phase of the inflammatory response, making it a marker of the systemic inflammatory response. When the body is stimulated by bacterial infection or bacteria or aseptic inflammatory stimuli such as atherosclerosis and cerebral infarction, CRP binds to lipoproteins, the complement system is activated, many inflammatory mediators are produced, and oxygen free radicals are released, causing damage to the vascular intima and increased vascular permeability and aggravating the systemic inflammatory response. Spearman analysis showed that CRP was positively correlated with AAC and an important indicator to alert the occurrence of AAC, so targeted prevention initiatives should be taken and close attention to gallbladder changes should be paid for patients with progressive elevation of CRP in the ICU.

(7) The APACHE-II score consists of the acute physiology score (APS), age, and chronic physiology score (CPS). It is thought that the severity of an acute disease can be determined by measuring the degree of irregularity in a number of physiological indicators, which is a commonly used index in the ICU to assess the severity of illness in ICU patients, with higher scores indicating greater severity of illness and needing more intense monitoring and treatment. In this study, the APACHE-II scores of both groups were high and generally above 15 points, and the overall baseline value was high; hence, the correlation was not significant.

(8) TPN and fasting will irritate patients' gastrointestinal tract, affect the peristalsis of the gastrointestinal tract, and then change the normal gallbladder movement rhythm, affecting bile discharge and causing congestion and edema of the gallbladder mucosa and a series of acute inflammatory reactions, which, combined with the use of sedative medications, can easily trigger obstruction at the common bile duct opening and increase the risk of AAC. Relevant animal experimental studies also confirmed that TPN and fasting easily induced cholestasis [22–25]. However, because of the diverse disease kinds of patients in each group and because patients with gastrointestinal disease usually had a longer period of TPN and fasting, significance was not presented in this study.

In conclusion, the APACHE-II score and time on TPN are not significantly correlated with the occurrence of AAC; and the amount of norepinephrine used, duration of ventilator used, white blood cell count, and serum CRP are positively correlated with AAC. Measuring the variations in the levels of various markers can signal the onset of AAC or reflect the state and prognosis, suggesting a possible application in clinic-based targeted prevention and treatment of AAC.

## Figures and Tables

**Table 1:** Between-group comparison of patients' general data.

Observation indicators	AAC group (*n* = 47)	Non-AAC group (*n* = 36)	*X* ^2^/*t*	*P*
Age (years)	63.15 ± 13.860	66.56 ± 15.230	1.064	0.290
BMI (kg/m^2^)	23.97 ± 3.120	24.06 ± 3.150	0.130	0.897
Length of hospital stay (d)	36.91 ± 46.300	22.97 ± 15.560	1.731	0.087
Gender			1.030	0.310
Male	30 (63.83)	19 (52.78)		
Female	17 (36.17)	17 (47.22)		
Smoking			0.001	0.973
Yes	9 (19.15)	7 (19.44)		
No	38 (80.85)	29 (80.56)		
Drinking			0.124	0.724
Yes	5 (10.64)	3 (8.33)		
No	42 (89.36)	33 (91.67)		
Nationality			0.578	0.447
Minorities	3 (6.38)	1 (2.78)		
Han	44 (93.62)	35 (97.22)		
Place of residence			0.218	0.640
Urban area	25 (53.19)	21 (58.33)		
Rural area	22 (46.81)	15 (41.67)		

**Table 2:** Between-group comparison of clinical data.

Observation indicator	AAC group	Non-AAC group	*X* ^2^/*t*	*P*
Shock time (d)	2.45 ± 1.07	1.11 ± 0.70	6.517	<0.001
Amount of norepinephrine used (*μ*g/kg)	32.53 ± 9.16	11.25 ± 4.10	12.966	<0.001
Duration of ventilator use (d)	8.81 ± 1.45	2.08 ± 0.64	25.951	<0.001
White blood cell count (×10^9^/L)	13.83 ± 4.34	7.55 ± 2.49	7.753	<0.001
CRP amount (mg/L)	105.40 ± 10.51	30.10 ± 6.81	37.370	<0.001
APACHE-II score	23.55 ± 5.03	18.69 ± 5.66	4.131	<0.001
Duration of sedative medication use (d)	6.83 ± 2.13	3.11 ± 0.97	9.725	<0.001
Time on TPN (d)	3.13 ± 1.23	2.64 ± 1.08	1.895	0.062
Fasting time (d)	4.15 ± 1.60	3.53 ± 1.26	1.914	0.059

**Table 3:** Spearman's correlation.

Test variable	*N*	Correlation coefficient	Sig. (two-sided)
Amount of norepinephrine used (*μ*g/kg)	83	0.827^∗^	0.000
Duration of ventilator use (d)	83	0.870^∗^	0.000
White blood cell count (×10^9^/L)	83	0.661^∗^	0.000
CRP amount (mg/L)	83	0.858^∗^	0.000

Note: ∗ denoted significant correlation at a confidence level (two-sided) of 0.001.

## Data Availability

Data to support the findings of this study is available on reasonable request from the corresponding author.
